The article "Smartphone GPS accuracy study in an urban environment" was published in 2019. Journal: PLoS One.

# Smartphone GPS accuracy study in an urban environment

**DOI:** 10.1371/journal.pone.0219890

**Published:** 2019-07-18

**Authors:** Krista Merry, Pete Bettinger

**Affiliations:** Warnell School of Forestry and Natural Resources, University of Georgia, Athens, GA, United States of America; National University of Singapore, SINGAPORE

## Abstract

An iPhone 6 using the Avenza software for capturing horizontal positions was employed to understand relative positional accuracy in an urban environment, during two seasons of the year, two times of day, and two perceived WiFi usage periods. On average, time of year did not seem to influence the average error observed in horizontal positions when GPS-only (no WiFi) capability was enabled, nor when WiFi was enabled. Observations of average horizontal position error only seemed to improve with time of day (afternoon) during the leaf-off season. During each season and during each time of day, horizontal position error seemed to improve in general during perceived high WiFi usage periods (when more people were present). Overall average horizontal position accuracy of the iPhone 6 (7–13 m) is consistent with the general accuracy levels observed of recreation-grade GPS receivers in potential high multi-path environments.

## Introduction

Smartphones have become ubiquitous tools of the human race, as millions of people now go about their days with small GPS-capable computers in their hands or pockets. The majority of current research involving smartphone GPS capabilities focuses on transportation or directional uses [1, 2, 3, 4], patterns of human movement [5, 6, 7], and health tracking [8, 9, 10]. Two interests of society involve (a) whether the accuracy is sufficient to enable them to be a reasonable substitute for more expensive commercially available mapping devices, and similarly (b) to what grade of receiver (consumer or mapping) could smartphones be a reasonable substitute. Much of what we do (navigate) or produce (map) is contingent on the level of horizontal position accuracy under conditions which GPS data is being collected. For example, a smartphone may not be the best option for collecting mappable information in predominantly forested conditions, but may be reliable enough for data collection purposes in urban environments. While the expectations for GPS data quality using an iPhone should not be assumed comparable to the quality of data collected with a mapping-grade or survey-grade GPS receiver, here we attempt to assess whether they can serve as a reasonable alternative and to measure what sort of error, both in distance and in direction, to expect. Therefore, the objective of this research was to assess the accuracy of the iPhone 6 GPS capabilities under various conditions. Specifically, this study is unique in the collection of static horizontal position data incorporating seasonal variability, level of human activity on the WiFi network, and urban forest conditions, and in assessing the role WiFi plays in GPS data collection accuracy.

The article "Smartphone GPS accuracy study in an urban environment" was published in 2019. Journal: PLoS One.

### Previous research

Modern smartphones are equipped with Assisted GPS (A-GPS) capability. A-GPS uses smartphone networks in combination with a GPS antenna to increase the speed of determining or fixing position [11]. A-GPS precludes the need of a warm-up period required for traditional GPS units [12]. However, data collected using A-GPS is less accurate than traditional GPS receivers [13, 14, 15]. Location based services (LBS) allow one to access spatial positioning on a phone via cellular networks [16]. Depending on the user’s phone settings, LBS are activated when permitted applications (apps) are in use (e.g., while using map apps). With the convenience and ease of use of the GPS capabilities of smartphone devices, it seems important to assess their accuracy, so when used for data collection purposes the relative accuracy of positions determined can be understood. There are numerous apps available to assist with GPS data collection. These allow the user to collect waypoints by simply tapping the screen of the phone. Depending on the app, a person can add their own basemap, interact with imagery provided by the app developer, and export saved positions from the app for use in other spatial software packages. A smartphone used in combination with an appropriate app can provide similar functionality as a basic recreation-grade GPS unit (e.g., Garmin, Magellan, etc.).

Mixed results can be found in the literature concerning the accuracy of smartphone GPS services. In a rather early study, using GPS enabled iPhones, iPods, an iPad and an app used by an insurance company in Switzerland, von Watzdorf and Michahelles [17] found average accuracy of location information between 108 and 655 m. More recently, the accuracy of static horizontal positions captured by a GPS-enabled phone was found to be around 20 m in one study [18]. This level of accuracy is most often influenced by landscape characteristics and the number of available satellites commonly leading to multipath errors. Multipath errors are the result of satellite signals bouncing off landscape features like buildings, trees, or the ground before entering the device. In another case, Menard et al. [19] found, in testing GPS accuracy across three different smartphone brands, that iPhone 4 determined approximately 98% of its GPS points within 10 m of true positions and approximately 59% within 5 m. When access to a WiFi network is available, that network is composed of access points that are used to help identify location [14], as a WiFi access point can emit its signal hundreds of meters. However, the number of WiFi access points available may have no impact on positional accuracy [20], contradicting early research that indicated accuracy might improve with increased access point availability [21]. Miluzzo et al. [22] conducted GPS data collection on the campus of Dartmouth College and determined that with a deterioration of smartphone service coverage and WiFi accessibility, accuracy also declined.

The article "Smartphone GPS accuracy study in an urban environment" was published in 2019. Journal: PLoS One.

In addition to the previously-noted studies, Zandbergen [14] found the average horizontal position error of an Apple iPhone 3G to be around 10 m, and Garnett and Stewart [23] found the average error for GPS points collected with Apple iPhone 4S to be around 6.5 m. Similar to the methodology presented in our study, Garnett and Stewart [23] sought to determine whether time of day impacted positional accuracy. Using three collection periods, early morning, mid-day, and late afternoon, they found that the first and second collection periods had no significant impact on horizontal position accuracy. They also noted no impact of weather conditions on positional accuracy. While the accuracy was higher for the Garmin GPS units, the iPhone was comparable overall in open areas and areas with lower building heights. Through the incorporation of a differential correction method to data collected on an Android smartphone Yoon et al. [24] reduced positional error down to 1 m during both static and dynamic data collection. In comparing a Garmin GPSMap 66 and an Android phone, Lachapell et al. [25] tested the GPS data collection capabilities under several different conditions including on a rooftop of a building, an urban canyon, indoors, and in a car. They found a reduction in multipath issues using the GPS receiver compared to the smartphone. The Garmin GPSMap 66 had a root mean square error (RMSE) below 1 m. Data collection in the vehicle using the Garmin unit again resulted in reduced multipath error. Modsching et al. [26] also noted that the presence of multi-story buildings can decrease the accuracy of horizontal determined positions, due to use of degraded signals in order to generate position fixes within urban canyons. Using a HTC G1 Dream and a Trimble Juno SB, Klimaszewski-Patterson [27] also assessed differences in accuracy between a smartphone and traditional GPS receiver. Using two different apps for GPS data collection, the residual error was lower when using the smartphone.

In contrast to the study of smartphones, more research has been conducted on the accuracy of traditional GPS receivers under forested conditions. Wing et al. [28] investigated the accuracy of several consumer-grade receivers across different forest canopy conditions (closed canopy dense forest, 40–50% canopy cover of a young Douglas-fir (*Pseudotsuga menziesii*) stand, and an area with no canopy cover). The average error for GPS collection ranged between 1 and 4 m in open areas, between approximately 1 and 7 m under a moderately dense canopy, and approximately 3 and 11 m under a closed forest canopy. In each forest condition, the average error was less than the manufacture’s assessment of 15 to 20 m accuracy. Within a dense Douglas-fir and western hemlock (*Tsuga heterophylla*) forest in Oregon, Wing and Eklund [29], measured comparable average positional accuracy between 5 and 9 m using a mapping-grade GPS receiver and between 5 and 12 m accuracy using a consumer-grade receiver following differential correction. Over a year’s worth of data collection, Bettinger and Fei [30] evaluated the accuracy of a Garmin Oregon 300 GPS receiver. Data collection occurred under varying forest conditions, within a hardwood stand and two pine stands with differing age classes, and nearly daily over the course of a year. Horizontal position accuracy (about 6–11 m) was not impacted by environmental conditions like temperature and relative humidity but varied significantly across forest stand types.

The article "Smartphone GPS accuracy study in an urban environment" was published in 2019. Journal: PLoS One.

In a mixed deciduous-coniferous forest, Tomaštík et al. [31] evaluated horizontal positional accuracy of three cellphones (ZTE Blade, LG G2, and Sony M4 Aqua), a tablet (Lenovo Yoga 8), a survey-grade GPS receiver and mapping-grade GPS receiver. Over the course of a leaf-on and leaf-off period, GPS data was collected at 74 points in a forested area at varying ages and density. Additionally, seventeen points were collected in an open meadow. For the three smartphones, average horizontal positional error ranged from 6.74 to 11.45 m in leaf-on conditions, from 4.51 to 6.72 m in leaf-off conditions, and from 1.90 to 2.36 in the open meadow.

## Materials and methods

### Study area

The University of Georgia, founded in 1785, is located in Athens, Georgia (USA). The nearly 800-acre campus serves as an educational facility for approximately 40,000 students. PAWS-Secure is the name of the WiFi network accessible to students, faculty, and staff, and this system is managed by the University’s Department of Enterprise Information Technology Services. The WiFi network is accessible in all buildings and green spaces on campus. The University of Georgia also has a system of survey monuments, benchmarks placed to identify surveyed points. Dispersed across the campus, the positions of these were surveyed and measured by the University Architects. The system contains 212 survey monuments of which six were selected for use in this study (Fig 1). Of the six monuments, five (Points 1–5) were established by surveyors in May 2015 and one was established in October 2003 (Point 6).

The article "Smartphone GPS accuracy study in an urban environment" was published in 2019. Journal: PLoS One.

**Fig 1:** Location of survey monuments used for sampling on the University of Georgia campus.

In an effort to describe the landscape surrounding each survey cap, a zone around each survey monument was created using a 30 m buffering process in a geographic information system (GIS). This 30 m buffer was chosen to represent an area twice as large as the largest mean error (14.15 m) from data collection across all survey monuments. A 2018 campus wide tree inventory provided by the University of Georgia’s Warnell School of Forestry and Natural Resources [32], was used to describe the number of trees that fell within the buffer around each survey monument using a point-in-polygon routine within GIS. A general description of the proximity (distance and direction) of each monument to nearby buildings was developed. Land cover within the buffer was delineated using USDA NAIP imagery (1 m spatial resolution) collected by the U.S. Department of Agriculture Farm Service Agency [33]. NAIP imagery is a digital ortho quarter quad (DOQQ) natural color image collected during the growing season across the continental U.S. At the time of this research, the most recently available imagery was collected in 2017.

Point (monument) 1 was located in the middle of a quad, with buildings on all sides and a network of sidewalks and grassy areas throughout. From Point 1, there is a three story building approximately 40 m to the northeast, approximately 60 m to the southeast is another three story building, approximately 40 m to the west is a four story building, and approximately 50 m to the southwest is a second four story building. Within the 30 m buffer, are thirty-nine trees that range in height between 2 and 22 m. Tree species within the buffer include fringe tree (*Chionanthus virginicus*), southern magnolia (*Magnolia grandiflora*), northern white cedar (*Thuja occidentalis*), tulip poplar (*Liriodendron tulipifera*), Chinese elm (*Ulmus parviflora*), willow oak (*Quercus phellos*), and red maple (*Acer rubrum*). Land cover within the 30 m was dominated by trees (30%), grass (37%), and sidewalks (22%).

Point 2 was located in a relatively open area, at the convergence of multiple walkways and adjacent to a road. The land cover of the polygon buffer is 40% sidewalk and roadway, 28% tree cover, and 31% grass. From Point 2, there is a three story building approximately 35 m to the northeast from the monument. Around 50 m from the monument to the northwest is a two story building, and 45 m to the southeast is a three story building. Within the 30 m sample buffer, there are thirty-three trees ranging in height from 2 to 23 m tall. The tree species included shortleaf pine (*Pinus echinata*), eastern redcedar (*Juniperus virginiana*), flowering dogwood (*Cornus florida*), water oak (*Quercus nigra*), willow oak, swamp chestnut oak (*Quercus michauxii*), red maple, and eastern redbud (*Cercis canadensis*).

The article "Smartphone GPS accuracy study in an urban environment" was published in 2019. Journal: PLoS One.

Point 3 was located at the intersection of two streets and approximately 30 m from a three story building, the monument is located in close proximity (approximately 3 m) to an 18 m tall overcup oak (*Quercus lyrata*). An additional 24 m tall overcup oak is approximately 15 m from the monument. In total there are eight trees within the 30 m sample buffer. Other species include nuttall oak (*Quercus nutallii*) and pin oak (*Quercus palustris*). Heights of the trees here range from 2 m to 14 m. The monument is also approximately 120 m from the university’s basketball coliseum. The land cover near the survey marker is dominated by a combination of sidewalks, roadways, and a parking lot (44%). Nearly one-third of the buffer contained tree cover (29%) and low vegetation like small shrubs (24%).

Point 4 was located at an intersection of two streets. The dominant land cover surrounding the survey monument is comprised of sidewalk and roadway (58%). Both grassy areas (22%) and tree cover (16%) were in close proximity to the sample point along with a minimal amount of low vegetation (4%). There were two trees, live oak (*Quercus virginiana*) and Yoshino cherry (*Prunus x yedoensis*), within the 30 m sample buffer around this monument ranging in height between 6 m and 14 m. Approximately 40 m to the north of the monument is a three story building. To the southeast, approximately 35 m from the monument, is a two story building.

Point 5 was located in a sidewalk adjacent to a street. Within the 30 m buffer around this monument, there are seventeen trees ranging in height from 2 to 30 m. The monument is located within 10 m of the largest tree in the sample with the tree crown extending over the monument during the leaf-on period. Tree species around this monument include pin oak, Nellie Stevens holly (*Ilex ‘Nellie R*. *Stevens’*), trident maple (*Acer buercerianum*), Texas redbud (*Cercis texensis*), Okame cherry (*Prunus x incamp ‘Okame’*), laurel oak (*Quercus laurifolia*), water oak, and pin oak. The majority of the land cover near the point was tree cover (47%) in addition to grassy areas (22%), sidewalks and roadways (17%), and a small amount of low vegetation (6%), and building (8%).

The article "Smartphone GPS accuracy study in an urban environment" was published in 2019. Journal: PLoS One.

Point 6 was located inside a parking lot median. Only 6% of the area in proximity to the survey monument is comprised of low vegetation and grassy areas. The predominant land cover is sidewalks and roadways (52%) and tree cover (36%). The closest building to the monument is approximately 30 m away, and the building is three stories tall. Within the 30 m sample buffer around this monument, there are fifty-seven trees, including eastern red cedars, two willow oaks, eighteen flowering dogwoods, slash pine (*Pinus elliotti*), willow oak, tulip poplar, European hornbeam (*Carpinus betulus*), and a fringe tree, which range in height from 2 to 20 m.

### Sampling design

A static horizontal position was recorded at each survey cap during one trip using LBS and the Avenza Maps app (https://www.avenza.com/avenza-maps/) on an iPhone 6. One trip entailed visiting each of the six points once in a clockwise or counter-clockwise order, as opposed to zig-zagging from point to point. For instance, if a trip began at Point 1 the next point visited would either be Point 4 or Point 2. Similarly, if the starting point for a trip was Point 5, the next point visited would be either Point 6 or Point 3. In order to randomize the sampling process, the starting point of each trip was randomized along with the direction of travel (clockwise or counter-clockwise). Trips were also separated by the time of day for sample collection. Samples were classified as morning (AM) samples collected between 8:00 AM EST and 11:59 AM eastern (USA) standard time, and afternoon (PM) samples collected between 12:00 PM EST and 5:00 PM. The timing of trips was divided into high and low activity times with respect to human activity on campus. High activity included days when classes were in session. Low activity included days when classes were not in session (weekends, holidays, spring break) or during the summer when the number of students taking classes was quite lower. Every effort was made to avoid collecting data when major sporting events occurred during what would normally be classified as low activity sampling periods. Finally, samples were collected during leaf-on and leaf-off periods. All leaf-on GPS collection was conducted between May 2017 and November 2017. All leaf-off GPS collection was conducted during two time periods: 1) from December 2016 to March 2017 and 2) March 2018. For the second time period, all data collection was completed during the month of March. During each data collection period, each point was visited 20 times. In total, there were eight separate data collection periods:

Period 1: High AM Leaf-on
Period 2: High PM Leaf-on
Period 3: Low AM Leaf-on
Period 4: Low PM Leaf-on
Period 5: High AM Leaf-off
Period 6: High PM Leaf-off
Period 7: Low AM Leaf-off
Period 8: Low PM Leaf-off

Using a unipod and a level, the phone was positioned over each survey cap, with the data collector oriented to face north (Fig 2). The phone was approximately three feet above the ground and was held away from the data collector's body during the data collection process. A block of wood was placed on the top of the unipod to aid in maintaining consistent positioning of the phone during data collection. Because of the design of the phone and in an effort to position the GPS and WiFi antennas as closely as possible to the true surveyed position during the data collection process, the phone was held in two different positions. At the top of the phone is both a 5 GHz antenna along with 2 GHz GPS / WiFi antenna. At the bottom of the phone is an additional WiFi antenna. When GPS-only sampling was conducted, the phone was held horizontally with the top half of the phone positioned over the survey monument. When WiFi sampling was performed, nearly three-quarters of the phone position was adjusted so that the middle of the phone was over the monument, since the two WiFi antennas are located on either end of the phone. For consistency, a piece of electrical tape was placed on the back of the phone approximately 5 cm from the top of the phone to mark where the phone should be positioned for GPS-only collection and another mark approximately 3 cm from the bottom of the phone for WiFi sampling. At each point, two GPS points were collected. For the first point collected, the phone’s WiFi capability was disabled. After the collection of the first point, the WiFi was enabled and two minutes were allowed to pass before the second data point was collected.

The article "Smartphone GPS accuracy study in an urban environment" was published in 2019. Journal: PLoS One.

**Fig 2:** a) Unipod, b) level, and c) survey cap.

A total of 160 trips were completed around the test course. During the leaf-on period, 476 total horizontal positions were collected. There were four instances where, during a trip, data collection was not possible at Points 1 and 4 due to construction vehicles parked over the monuments. During the leaf-off period, there was one instance where a data point was not collected at Point 1 due to a vehicle being parked over a monument, therefore 479 data points were collected during the leaf-off period. During the leaf-on period, there were 29 instances where the WiFi capability was enabled for WiFi data collection but no WiFi connection was observed during the two-minute period following GPS-only point collection. Whether a WiFi connection was made was based on whether or not the WiFi status icon was activated on the phone interface. In keeping with the pre-determined data collection protocol, a waypoint was collected and a note was made that no WiFi connection had been made. Similarly, during the leaf-off data collection period, there were 38 instances where a WiFi connection was not evident. Across both leaf-on and leaf-off data collection periods, this situation most often occurred at Point 6, where 11 visits during leaf-off and 18 visits during leaf-on the WiFi status icon on the phone screen was not activated.

After the completion of each trip, the horizontal positions collected were exported from the phone as a .KML file and then converted to point shapefiles for use in GIS. Data were then converted from latitude / longitude to UTM NAD83 UTM Zone 17 N allowing analysis to be conducted in the same units (meters) as the data associated with the monuments. One aim of this research endeavor was to determine whether using WiFi affected the horizontal position accuracy of the GPS data. Additionally, we were interested in whether an increased number of potential WiFi-users on campus had any impact on the horizontal position accuracy during data collection. Finally, we wanted to quantify the amount of horizontal position error a user could expect when collecting GPS points in an urban environment using an iPhone 6. For this, Euclidean distances were determined between the monument position and the location of each horizontal position recorded.

### Statistical tests

Statistical tests were employed to determine whether positional error from GPS-only and WiFi-enabled data were significantly different. Using nineteen collection categories (Table 1), the following hypotheses were tested:

H_o_: The horizontal position errors of the GPS-only and WiFi data are not distributed differently.
H_1_: The horizontal position errors of the GPS-only and WiFi data are distributed differently.

**Table 1:** Outcomes of GPS-only and WiFi-enabled comparisons using the Mann-Whitney Test (R = reject null hypothesis, FR = failed to reject null hypothesis, p<0.05)).

Collection Period	Point 1	Point 2	Point 3	Point 4	Point 5	Point 6	All
ALL	FR (p = 0.254)	FR (p = 0.776)	FR (p = 0.359)	FR (p = 0.334)	FR (p = 0.094)	FR (p = 0.543)	R (p = 0.042)
AM	FR (p = 0.491)	FR (p = 0.612)	FR (p = 0.929)	FR (p = 0.204)	FR (p = 0.325)	FR (p = 0.393)	R (p = 0.028)
PM	FR (p = 0.391)	FR (p = 0.997)	FR (p = 0.184)	FR (p = 0.970)	FR (p = 0.165)	FR (p = 0.992)	FR (p = 0.480)
HIGH	R (p = 0.014)	FR (p = 0.425)	FR (p = 0.396)	FR (p = 0.787)	FR (p = 0.242)	FR (p = 0.489)	R (p = 0.373)
LOW	FR (p = 0.504)	FR (p = 0.622)	FR (p = 0.634)	FR (p = 0.221)	FR (p = 0.213)	FR (p = 0.879)	FR (p = 0.395)
Leaf-On	FR (p = 0.428)	FR (p = 0.318)	FR (p = 0.234)	FR (p = 0.785)	FR (p = 0.716)	FR (p = 0.484)	FR (p = 0.826)
Leaf-Off	R (p = 0.023)	FR (p = 0.168)	FR (p = 0.933)	FR (p = 0.310)	R (p = 0.028)	FR (p = 0.974)	R (p = 0.004)
HIGH AM	R (p = 0.028)	FR (p = 0.447)	FR (p = 0.814)	FR (p = 0.676)	FR (p = 0.358)	FR (p = 0.381)	R (p = 0.024)
HIGH PM	FR (p = 0.235)	FR (p = 0.729)	FR (p = 0.361)	FR (p = 0.981)	FR (p = 0.436)	FR (p = 0.992)	FR (p = 0.509)
LOW AM	FR (p = 0.220)	FR (p = 0.755)	FR (p = 0.755)	FR (p = 0.145)	FR (p = 0.577)	FR (p = 0.840)	FR (p = 0.382)
LOW PM	FR (p = 0.863)	FR (p = 0.637)	FR (p = 0.331)	FR (p = 0.740)	FR (p = 0.225)	FR (p = 0.985)	FR (p = 0.677)
HIGH AM Leaf-On	FR (p = 0.293)	FR (p = 0.862)	FR (p = 0.820)	FR (p = 0.478)	FR (p = 0.327)	FR (p = 0.659)	FR (p = 0.224)
HIGH PM Leaf-On	FR (p = 0.659)	FR (p = 0.883)	FR (p = 0.429)	FR (p = 0.659)	FR (p = 0.758)	FR (p = 0.904)	FR (p = 0.478)
LOW AM Leaf-On	R (p = 0.021)	FR (p = 0.314)	FR (p = 0.445)	FR (p = 0.341)	FR (p = 1.011)	FR (p = 0.883)	FR (p = 0.650)
LOW PM Leaf-On	FR (p = 0.314)	FR (p = 0.602)	FR (p = 0.461)	FR (p = 0.221)	FR (p = 0.060)	FR (p = 0.478)	FR (p = 0.549)
HIGH AM Leaf-Off	R (p = 0.049)	FR (p = 0.253)	FR (p = 0.698)	FR (p = 0.989)	FR (p = 0.779)	FR (p = 0.355)	FR (p = 0.052)
HIGH PM Leaf-Off	R (p = 0.038)	FR (p = 0.512)	FR (p = 0.698)	FR (p = 0.841)	FR (p = 0.114)	FR (p = 0.968)	FR (p = 0.133)
LOW AM Leaf-Off	FR (p = 0.947)	FR (p = 0.620)	FR (p = 0.192)	FR (p = 0.311)	FR (p = 0.478)	FR (p = 0.883)	FR (p = 0.142)
LOW PM Leaf-Off	FR (p = 0.314)	FR (p = 0.602)	FR (p = 0.461)	FR (p = 0.221)	FR (p = 0.060)	FR (p = 0.369)	FR (p = 0.236)

The sets of static horizontal position errors of the nineteen different data collection scenarios were tested for normality using a Shapiro-Wilk test. We found that the sets of data were generally not normally distributed. Therefore, a non-parametric test for statistical significance was required for statistical analysis [34]. Using the Mann-Whitney test is common when assessing GPS accuracy [35, 36, 37, 38, 39, 40]. The Mann-Whitney test was implemented at a 95% confidence level to test the null hypothesis that the static horizontal position error collected during GPS-only data collection was not significantly different than the static horizontal position error collected when WiFi was enabled. Further, to describe the positional error, descriptive statistics including minimum and maximum error, and the RMSE of the horizontal position error were calculated for data collected at each sample point and under each of the eight data collection periods. RMSE illustrates the error between the known location (the survey monument) and the collected location (waypoint). Specifically, RMSE is the square root of the average set of squared distances between a known location and the location recorded during data collection. RMSE is a common measurement of horizontal position accuracy in GPS research [14, 30, 31, 41, 42]. In an attempt to identify what may be causing the horizontal position error, Pearson’s correlation coefficient was used to determine whether land cover was correlated with the horizontal position accuracy of data. Pearson’s correlation coefficient measures the association between two variables expressed based on a value ranging between -1 (negative correlation), 0 (no correlation), and +1 (positive correlation) [43].

The article "Smartphone GPS accuracy study in an urban environment" was published in 2019. Journal: PLoS One.

Finally, local weather data variables were compiled for the period of time during which the sampling cycle was completed. Meteorological data was recorded for the time period of each trip using reports from nearby Athens Ben Epps Airport. Weather variables included air temperature (°F), relative humidity (%), barometric pressure (inches), wind speed (mph), and condition (clear, partly cloudy, mostly cloudy, scattered clouds, overcast). Pearson's correlation coefficient was used to determine whether these weather characteristics were correlated with the horizontal position accuracy of the data collected. Separately, a multivariate regression analysis was performed to identify the influence of weather conditions on positional error. Regression analysis was chosen because it allowed for an analytical method for incorporating categorical data. To do so, each weather condition was converted into a dummy variable containing values of 0 (the weather condition was not recorded at the time of data collection) or 1 (the weather condition was recorded at the time of data collection). Each weather condition served as an independent variable in the regression analysis with a total of 5 independent variables.

## Results

In examining all horizontal position error derived during the GPS-only data collection effort, the minimum positional error was 0.05 m compared to a maximum error of 99.7 m. The RMSE for all data collected with the iPhone in GPS-only mode was about 9.9 m. On average, time of year did not seem to influence the average error observed in horizontal positions when GPS-only capability was assumed. In terms of overall performance, some improvement was observed in RMSE during the leaf-off period, but not in every case (e.g., High AM). Points 3 and 5 seemed to have the highest RMSE during the leaf-on period, and were joined by Point 1 during the leaf-off period (Table 2). It should be noted that relatively large confidence intervals were also derived from the sample data, indicating significant variability in the observed positional errors. The RMSE was generally lowest at Points 2 and 6, which were in relatively open areas, thus there is an assumed reduction in multipath error. The overall average horizontal position error was worst during the Low AM data collection period over both seasons. The single maximum horizontal position error observation was observed at Point 4 (about 100 m), and is likely an outlier as the next largest single observation of horizontal position error was approximately 30 m (Table 3). The minimum horizontal position error from a single observation, across all points and seasons, fell below 1 m at least once in 20 of the 48 cases (6 points, 8 data collection periods) and fell below 2 m at least once in 39 of the 48 cases (Table 3).

The article "Smartphone GPS accuracy study in an urban environment" was published in 2019. Journal: PLoS One.

**Table 2:** RMSE and 95% confidence intervals for horizontal positions collected with GPS only.

		Leaf-On				Leaf-Off		
		RMSE (m) (95% ±CI)				RMSE (m) (95% ±CI)		
	*High AM*	*High PM*	*Low AM*	*Low PM*	*High AM*	*High PM*	*Low AM*	*Low PM*
	(Period 1)	(Period 2)	(Period 3)	(Period 4)	(Period 5)	(Period 6)	(Period 7)	(Period 8)
Point 1	7.52 (±1.96)	7.36 (±1.30)	10.94 (±1.81)	8.91 (±1.49)	9.09 (±2.89)	7.56 (±2.28)	13.66 (±3.93)	13.73 (±4.95)
Point 2	2.60 (±0.50)	5.10 (±1.30)	3.87 (±0.53)	5.00 (±1.27)	5.86 (±1.74)	2.64 (±0.60)	3.73 (±0.82)	2.36 (±0.43)
Point 3	11.69 (±3.36)	9.27 (±1.86)	12.29 (±2.35)	12.42 (±2.84)	10.47 (±2.16)	10.58 (±3.09)	13.22 (±4.50)	13.42 (±3.87)
Point 4	5.76 (±1.57)	8.63 (±1.69)	22.84 (±9.41)	8.14 (±1.98)	9.40 (±2.76)	6.79 (±1.95)	7.63 (±2.31)	6.46 (±2.06)
Point 5	9.39 (±1.96)	15.98 (±5.02)	13.50 (±3.88)	14.82 (±3.81)	18.92 (±5.64)	11.37 (±3.07)	16.27 (±4.62)	11.04 (±3.88)
Point 6	2.97 (±0.73)	4.30 (±0.82)	4.71 (±0.80)	6.30 (±1.71)	3.30 (±0.73)	2.78 (±0.74)	2.81 (±0.66)	3.23 (±0.77)
Overall	7.42 (±0.90)	9.07 (±1.07)	12.99 (±1.82)	9.89 (±1.08)	10.67 (±1.39)	7.73 (±0.99)	10.87 (±1.47)	9.56 (±1.36)

**Table 3:** Minimum and maximum horizontal position error by collection period using GPS only.

		Leaf-On				Leaf-Off		
		Min / Max (m)				Min / Max (m)		
	*High AM*	*High PM*	*Low AM*	*Low PM*	*High AM*	*High PM*	*Low AM*	*Low PM*
	(Period 1)	(Period 2)	(Period 3)	(Period 4)	(Period 5)	(Period 6)	(Period 7)	(Period 8)
Point 1	1.37 / 17.82	1.93 / 12.76	2.14 / 23.50	1.82 / 16.46	0.78 / 28.06	0.20 / 20.55	1.80 / 37.52	0.26 / 40.80
Point 2	0.72 / 4.51	1.06 / 14.04	1.90 / 6.41	1.59 / 12.02	1.47 / 17.26	0.40 / 5.24	0.91 / 8.14	0.54 / 3.98
Point 3	2.71 / 30.26	2.50 / 16.34	3.44 / 22.66	0.97 / 23.79	2.97 / 20.49	0.55 / 24.58	1.03 / 37.58	1.94 / 32.71
Point 4	0.52 / 15.68	2.60 / 15.53	1.00 / 99.67	0.88 / 15.44	1.28 / 28.02	0.63 / 19.86	1.35 / 18.26	1.02 / 18.41
Point 5	2.70 / 19.06	1.13 / 41.83	0.70 / 29.85	1.74 / 33.97	1.85 / 42.86	2.15 / 23.84	2.35 / 35.01	0.05 / 38.89
Point 6	0.63 / 6.46	1.76 / 8.21	1.52 / 8.27	0.31 / 13.66	0.31 / 6.00	0.22 / 1.08	0.85 / 5.49	0.60 / 8.15

On average, time of year also did not seem to influence the average error observed in horizontal positions when WiFi capability was enabled. Again, Points 3 and 5 seemed to have the highest RMSE during the leaf-on period, joined by Point 1 during the leaf-off period (Table 4). And as with the GPS-only data, relatively large confidence intervals were derived from the sample data at these points, indicating significant variability in the observed positional errors. Further, the RMSE was again generally lowest at Points 2 and 6, which were in relatively open areas, thus there is an assumed reduction in multipath error. In contrast to the GPS-only results, the overall RMSE was highest during the High AM data collection periods during the leaf-off season. The single maximum horizontal position error observation was observed at Point 5 (about 39 m) when WiFi was enabled (Table 5), and the single minimum horizontal position error observation was observed at Point 6 (about 11 cm). The minimum horizontal position error from a single observation, across all points and seasons, fell below 1 m in 15 of the 48 cases, and fell below 2 m in 35 of the 48 cases (Table 5).

The article "Smartphone GPS accuracy study in an urban environment" was published in 2019. Journal: PLoS One.

**Table 4:** RMSE and 95% confidence intervals for horizontal positions collected with WiFi enabled.

		Leaf-On				Leaf-Off		
		RMSE (m) (95% ±CI)				RMSE (m) (95% ±CI)		
	*High AM*	*High PM*	*Low AM*	*Low PM*	*High AM*	*High PM*	*Low AM*	*Low PM*
	(Period 1)	(Period 2)	(Period 3)	(Period 4)	(Period 5)	(Period 6)	(Period 7)	(Period 8)
Point 1	8.22 (±1.73)	6.39 (±0.96)	10.21 (±2.39)	8.78 (±1.80)	11.69 (±3.01)	9.01 (±2.20)	12.43 (±3.52)	11.30 (±3.60)
Point 2	2.85 (±0.62)	3.92 (±0.90)	3.50 (±0.55)	7.29 (±2.61)	7.82 (±2.22)	2.91 (±0.59)	3.89 (±0.80)	2.64 (±0.51)
Point 3	8.52 (±1.72)	7.42 (±1.25)	11.06 (±2.27)	10.48 (±2.37)	9.88 (±2.02)	6.47 (±1.26)	11.73 (±3.25)	9.42 (±2.41)
Point 4	5.43 (±1.16)	7.85 (±1.45)	7.12 (±1.77)	6.28 (±1.26)	9.32 (±2.68)	6.34 (±1.54)	7.67 (±2.01)	6.82 (±2.03)
Point 5	11.85 (±2.65)	13.33 (±4.28)	13.01 (±3.65)	14.97 (±3.55)	15.46 (±3.88)	11.38 (±2.13)	15.87 (±3.81)	11.68 (±3.45)
Point 6	6.56 (±2.34)	4.39 (±0.90)	5.68 (±1.39)	6.78 (±1.79)	5.82 (±1.65)	4.26 (±1.50)	4.11 (±1.28)	2.59 (±0.58)
Overall	7.75 (±0.87)	7.85 (±0.90)	9.05 (±1.00)	9.62 (±1.08)	10.45 (±1.17)	7.30 (±0.81)	10.30 (±1.27)	8.30 (±1.08)

**Table 5:** Minimum and maximum distance horizontal position error by collection period using WiFi.

		Leaf-On				Leaf-Off		
		Min / Max (m)				Min / Max (m)		
	*High AM*	*High PM*	*Low AM*	*Low PM*	*High AM*	*High PM*	*Low AM*	*Low PM*
	(Period 1)	(Period 2)	(Period 3)	(Period 4)	(Period 5)	(Period 6)	(Period 7)	(Period 8)
Point 1	2.45 / 14.97	1.58 / 9.75	1.90 / 29.28	1.51 / 15.11	1.77 / 24.79	1.92 / 18.91	1.80 / 32.29	1.57 / 33.05
Point 2	0.55 / 5.94	0.90 / 8.82	0.71 / 5.55	1.26 / 28.20	0.62 / 19.84	0.59 / 5.54	1.03 / 9.29	0.27 / 4.39
Point 3	2.71 / 16.60	2.20 / 12.11	2.18 / 28.72	1.84 / 23.84	2.86 / 18.52	2.18 / 10.87	2.14 / 33.02	1.86 / 20.61
Point 4	1.53 / 10.74	2.27 / 12.81	1.10 / 15.57	1.76 / 11.23	1.27 / 23.98	0.52 / 13.58	0.43 / 15.13	1.52 / 18.41
Point 5	2.14 / 22.68	1.13 / 38.62	0.44 / 22.53	1.36 / 29.53	2.07 / 32.64	2.80 / 21.73	3.24 / 31.79	1.75 / 36.75
Point 6	0.72 / 22.94	1.50 / 10.65	2.19 / 15.93	0.83 / 19.85	0.31 / 12.45	0.11 / 16.24	0.19 / 13.18	0.31 / 4.43

Across all of the combinations of data collection conditions examined, there were only 12 (out of 133) instances where the sets of horizontal position error were statistically significantly different (*p* < 0.05, Table 1). When considering all observations of horizontal position error during GPS-only data collection compared to all horizontal position error during WiFi data collection, the null hypothesis was rejected and therefore the data are statistically significantly different (*p* < 0.05). However, we could not reject the null hypothesis when only considering the data collected from a single sample point. The error was also statistically significantly different when considering all sets of observations of horizontal position error observed during AM, Leaf-off, and high data collection periods High AM and High PM (separately) data collection periods. Sample Point 1 was the only point where there were many instances of detection of significant differences among the GPS-only and WiFi-enabled data. While we cannot be completely certain what is causing the significant differences at this sample point, Point 1 is unique in that it is surrounded on each side by multistory buildings which may be increasing the positional error when GPS-only data was collected. However, each of these buildings house WiFi access points which may lead to a stronger WiFi signal at this point reducing the positional error when the WiFi is enabled.

The article "Smartphone GPS accuracy study in an urban environment" was published in 2019. Journal: PLoS One.

In examining the frequency of the error across all points, interesting patterns emerge (Fig 3). For instance, during GPS-only data collection, both Points 2 and 6 had no instances of error sampling. Similar to Point 1, the occurrence of error was mostly clustered in between 2 m and 20 m during GPS-only data collection. However, when WiFi was enabled, there were nearly twice as many occurrences of error (*n* = 76) between 5 and 10 m than any other error range. The error distributions at Point 4 and Point 5 were very similar between WiFi and GPS-only sampling with the majority of error falling between 2 to 10 m at Point 4 and ranging from 2 m to more than 20 m at Point 5. The frequency of horizontal position error at Point 6 was most prominent between the 0 and 2 m and 2 to 5 m ranges for both GPS-only and WiFi data collection.

**Fig 3:** Frequency distribution of GPS only and WiFi horizontal position error by five error classes.

In an effort to identify what might be causing the horizontal error, a correlation between the percent land cover within the 30 m sample buffer and the error was derived (Table 6). A moderate positive correlation between the building land cover class and horizontal positional error was found during GPS-only data collection indicating that an increased presence of buildings led to an increase in horizontal positional error. This correlation was more pronounced during WiFi-enabled data collection but still only moderately. Minor positive correlations were found between tree cover and low vegetation and error during both GPS-only and WiFi-enabled data collection. Additionally, a minor negative correlation was found between the percent land cover classified as sidewalks, roads, and parking lots and positional error.

**Table 6:** Pearson’s correlation coefficient results between percent land cover and GPS only and WiFi enabled data.

	Trees	Buildings	Grass	Low Veg.	Sidewalks / Roads /
					Parking Lots
	(%)	(%)	(%)	(%)	(%)
GPS-only	0.1249	0.3236	-0.0409	0.2148	-0.2218
WIFI-enabled	0.2133	0.4236	0.0102	0.1748	-0.3217

While understanding the amount of horizontal error between a survey monument and a position collected by the iPhone 6 is useful, knowing the predominant direction of that error may also be important. In examining the directional error, the angle between survey monuments and positions determined by the iPhone was calculated, and some general patterns emerged. For example, directional error at Point 1 using GPS-only data predominantly ranged in cardinal direction from south to north with a majority of directional error occurring in a west to northwest direction under all data collection conditions (Fig 4), yet during data collection Period 3, there was no dominant direction of error. When WiFi was enabled, the direction of error was comparable to GPS-only (Fig 5) but most pronounced from the west to northwest. At Point 2, there were several instances where there was no dominant direction of error during GPS-only data collection periods yet when considering data collected under all data collection conditions the error most often occurred from southwest to north. When WiFi was enabled, error typically occurred in a westerly pattern ranging from the west-southwest to north-northwest. GPS-only data collection at Point 3 revealed directional error predominantly ranging from west-northwest to the north-northeast. During two collection periods, Low AM leaf-on and Low PM leaf-on, there was no dominant directional error suggesting error was dispersed in all directions. During WiFi data collection, error during Period 1 and Period 3 were consistently in a northerly direction clustered between north-northwest and north-northeast, and in most other cases northwest to northeast. When WiFi was enabled at Point 4, the direction of error often ranged between south-southwest to north-northwest while error was more dispersed across the cardinal directions for GPS-only data. During GPS-only data collection at Point 5, the vast majority of data error in all data collection conditions fell between the cardinal directions of west-southwest and north. Similarly, when WiFi-enabled data collection occurred at Point 5, the majority of direction error fell between west-southwest and north-northwest. Conversely, at Point 6 when using GPS-only there were 5 different collection periods where there was no pronounced directional error, yet when directional error was pronounced, there was little consistency between data collection periods. When WiFi was enabled at this point, the directional error lacked a dominant direction.

The article "Smartphone GPS accuracy study in an urban environment" was published in 2019. Journal: PLoS One.

**Fig 4:** Rose diagrams illustrating directional error of data collected using GPS-only capabilities of an iPhone 6.

**Fig 5:** Rose diagrams illustrating directional error of data collected using WiFi enabled capabilities of an iPhone 6.

Finally, almost uniformly, there was generally weak to no correlation between horizontal position error of the positions determined by the iPhone, and temperature, barometric pressure, wind speed, and relative humidity during the data collection effort (Table 7). The results of the multivariate regression analysis indicated that there was no relationship between GPS-only positional error (adjusted R^2^ = -0.0009) and weather condition (i.e., clear, partly cloudy, etc). Similarly, when WiFi was enabled positional error was also not related (adjusted R^2^ = -0005) to current weather conditions.

**Table 7:** Pearson’s correlation coefficient results between weather conditions and GPS only and WiFi enabled data.

	Air	Barometric	Wind	Relative
	temperature	Pressure	speed	humidity
	(°F)	(inches)	(mph)	(%)
GPS-only	0.0256	0.0522	-0.0339	0.0514
WIFI-enabled	-0.0188	0.0666	-0.0264	0.0428

## Discussion

When considering the static horizontal position error from all data points collected, the error observed in GPS-only data was significantly different from the error observed in the WiFi- enabled data. Further, data collected in the morning, and data collected during high WiFi use periods also indicated that GPS-only data and WiFi-enabled data had significantly different levels of horizontal position error. During only the leaf-off season were similar significant differences observed between GPS-only and WiFi-enabled data. These observations, while not significant at every data collection point, suggest that on average, enabling the iPhone to use WiFi signals to augment the determination of horizontal positions will lead to higher quality positional information. While it was unclear how extensive the WiFi services were utilized by the iPhone, the opportunity to use these services affected positional accuracy. Interestingly, nearby buildings may have influenced the direction of error observed, due likely to multipathed signals from either the GPS satellite constellation or the WiFi signal emitting devices.

The article "Smartphone GPS accuracy study in an urban environment" was published in 2019. Journal: PLoS One.

One pattern became evident when interpreting the results for data collected when the WiFi was enabled: the average positional error was greater around Point 5 than all other test points, regardless of leaf-on or leaf-off conditions, and morning or afternoon data collection efforts, the error was most pronounced at this point. Some of this could likely be explained by multipath conditions or a simple deterioration in GPS signals. However, this survey monument was located across a two-lane street from a multistory hotel and convention center and under a large tree. Comparatively, Points 2 and 6 were frequently the data collection points with the lowest RMSE, particularly during WiFi data collection periods. During GPS-only collection, Point 6 had low positional error compared to data collected at other survey monuments. Each of these monuments (Points 2 and 6) were located in relatively open areas, and thus this may indicate that what plays the largest role in smartphone GPS data accuracy may be proximity to multistory structures, rather than increased activity on a nearby WiFi network or the presence of nearby trees. Further, our work has provided results that are similar to those provided by Garnett and Stewart [23], Weaver et al. [42] and others who have shown no correlation between atmospheric conditions and static horizontal position accuracy of low- to moderate-cost GPS receivers.

This observational study is one of the first of its kind to examine the positional accuracy of horizontal positions determined by a smartphone during high and low human activity, and during two different seasons of the year (influencing the amount and presence of nearby tree canopies). Many of the influential factors could not be closely controlled by the study team; therefore, numerous samples were collected over each survey monument during random times of the day to understand on average the level of positional error one might expect. While protocols for data collection seem reasonable (randomize the order of data collection, routinely collect data in the same manner at each monument, etc.), some of the uncontrollable aspects of the data collection process included the amount of human activity (high and low were all we could assume), and the status and condition of the WiFi network managed by the university. Persistent efforts were employed to acquire information on the status of the network during the data collection periods, yet we were unable to acquire metrics regarding the WiFi signal status around the test course due to the university not allowing us access to these metrics. As a result, our observations should reflect average performance of the smartphone under average WiFi operating conditions.

The article "Smartphone GPS accuracy study in an urban environment" was published in 2019. Journal: PLoS One.

This study could be complemented by further studies that focus on some of the limitations we observed. For example, we were unable to sufficiently understand why horizontal position accuracy improved during periods of time when WiFi usage was high. Given our lack of access to the technical specifications of the WiFi network, perhaps management of the network during high use periods contributed to this result. Additional research that incorporates a measurement of the strength of the WiFi signal at each sample point would be useful. Further, the results we observed were highly variable around each sample point, perhaps due to the heterogeneous nature of the urban environment (spatial arrangement of trees, buildings, etc.). A complementary study to better understand the impact of the spatial arrangement of features, similar to that of Bettinger and Merry [41] that was conducted in a forest, may further our understanding of these issues. To further investigate the role multipath plays in error, it would be useful to set up a device at each sample point and continuously collect data over a period of time and at specified time intervals. Here, the assumption is that the error would repeat as long as the surrounding landscape (buildings, trees, etc.) remained the same. And finally, as computing technology continues to evolve, continued observational and hypothesis-driven studies of smartphone accuracy in urban environments will be necessary to inform society of the potential practical and scientific uses of these hand-held positional and navigational devices. Specifically, a similar research endeavor using a newer smartphone with an improved GPS chip would be valuable.

The article "Smartphone GPS accuracy study in an urban environment" was published in 2019. Journal: PLoS One.

## Conclusions

The horizontal position error associated with GPS positions determined by a smartphone is often assumed negligible by ordinary users of the technology. However, as smartphones are used more often for data collection purposes, perhaps during crowd sourcing data collection exercises or the capture of positional information through various smartphone apps, this concern may need more attention. Our study has shown that the overall average horizontal position error of the iPhone 6 is in the 7–13 m range, depending on conditions, which is consistent with the general accuracy levels observed of recreation-grade GPS receivers in potential high multipath environments. It seemed in our study that the time of year did not influence the average horizontal position error observed when GPS-only parameters were assumed, or when WiFi was enabled. Our observations of average horizontal position error only seemed to improve with time of day (afternoon) during the leaf-off season. Interestingly, horizontal position error seemed to improve in general during perceived high WiFi usage periods (when more people were present) within each season and during each time of day most prominently in the afternoon. In general, directional error was consistent at each data collection point during both GPS-only and WiFi collection. The most pronounced instance of directional error occurred at Point 5 in a west to northwest direction. Data collection may have been subjected to multipath issues at some of the data collection points. We saw moderate correlation between the presence of buildings and positional error during both GPS-only and WiFi-enabled data collection. Finally, weather conditions had little to no influence on the accuracy of data collected.

## Supporting information

S1 Data Spreadsheet containing GPS data collected. (XLSX)

S2 Data Weather data associated with data collection. (XLSX)
